# Deferiprone−Resveratrol Hybrid, an Iron-Chelating Compound, Acts as an Antimalarial and Hepatoprotective Agent in *Plasmodium berghei*-Infected Mice

**DOI:** 10.1155/2022/3869337

**Published:** 2022-11-24

**Authors:** Hataichanok Chuljerm, Supawadee Maneekesorn, Chuchard Punsawad, Voravuth Somsak, Yongmin Ma, Jetsada Ruangsuriya, Somdet Srichairatanakool, Pimpisid Koonyosying

**Affiliations:** ^1^School of Allied Health Sciences, Walailak University, Nakhon Si Thammarat 80160, Thailand; ^2^School of Health Sciences Research, Research Institute for Health Sciences Chiang Mai University, Chiang Mai 50200, Thailand; ^3^Environmental and Occupational Health Sciences and Non Communicable Diseases Research Group (EOHS and NCD Research Group), Research Institute for Health Sciences Chiang Mai University, Chiang Mai 50200, Thailand; ^4^Faculty of Medical Technology, Nation University, Lampang 52000, Thailand; ^5^School of Medicine, Walailak University, Nakhon Si Thammarat 80160, Thailand; ^6^School of Pharmaceutical Sciences, Taizhou University, Zhejiang 318000, China; ^7^Department of Biochemistry, Faculty of Medicine Chiang Mai University, Chiang Mai 50200, Thailand

## Abstract

Free heme in plasma acts as a prooxidant; thus, it is bound to hemopexin and eliminated by the liver. High iron content in the liver can support *Plasmodium* growth and cause oxidative liver injury. Inversely, the withholding of excessive iron can inhibit this growth and protect the liver against malaria infection. This study examined the effects of a deferiprone-resveratrol (DFP-RVT) hybrid on malaria parasites and its relevant hepatoprotective properties. Mice were infected with *P. berghei*, gavage DFP-RVT, deferiprone (DFP), and pyrimethamine (PYR) for 8 consecutive days. Blood and liver parameters were then evaluated. The presence of blood-stage parasites was determined using the microscopic Giemsa staining method. Subsequently, plasma liver enzymes, heme, and concentrations of thiobarbituric acid-reactive substances (TBARS) were determined. The liver tissue was examined pathologically and heme and TBARS concentrations were then quantified. The results indicate that the suppression potency against *P. berghei* growth occurred as follows: PYR > DFP-RVT hybrid > DFP. Importantly, DFP-RVT significantly improved RBC size, restored alanine aminotransferase and alkaline activities, and increased heme and TBARS concentrations. The compound also reduced the liver weight index, heme, and TBARS concentrations significantly when compared to mice that were untreated. Our findings support the contention that the hepatoprotective effect of DFP-RVT is associated with parasite burden, iron depletion, and lipid peroxidation in the host.

## 1. Introduction

Malaria is a devastating disease that is caused by *Plasmodium* parasites and has been associated with significant rates of morbidity and mortality [1]. In cases of advanced infection, severe anemia can occur leading to organ dysfunction and conditions of hypoxia [2, 3]. Mammals encode the heme oxygenase (HO) gene that is known to synthesize the HO-1 enzyme to cleave the protoporphyrin rings of heme at the expense of O_2_ in releasing linear biliverdin, carbon monoxide, and Fe^2+^, which then bind to transferrin in the plasma or can be stored in ferritin in the liver. As lower eukaryotes, plasmodium parasites lack the HO needed to degrade toxic heme derived from the degradation of digested red blood cells (RBC) from hemoglobin (Hb); therefore, they must convert the heme into a nontoxic hemozoin/*β*−hematin [4, 5]. Consequently, liver damage, renal failure, and spleen enlargement are some of the harmful consequences. Critically, severe intra- and extra-vascular hemolysis will occur during erythrocytic malaria infection [6] depending upon the degree of the parasite load [7]. Accordingly, free Hb is released into the blood. It is subsequently bound to haptoglobin and removed by the liver. As a consequence, the ability of Hp to scavenge free Hb is overwhelmed [3, 8], while ferrous Hb in the blood is oxidized to ferric Hb (methemoglobin) which is then dissociated to heme and globin. Coincidently, hemopexin fails to remove excessive heme leading to increased heme concentrations in the plasma [8, 9]. Importantly, free heme is toxic to the body. It is known to catalyze the production of reactive oxygen species (ROS) via the Fenton reaction and cause both oxidative tissue damage and organ failure [10, 11].

Though several antimalarial drugs are available for the treatment of malaria, they have been associated with toxicity and a degree of resistance by the parasite [12, 13]. With regard to toxicity, prophylactic antimalarial drugs, such as amodiaquine, chloroquine, or pyrimethamine, may cause leucopenia and abnormal liver function [14, 15]. Evidently, one-third of malaria-infected patients have experienced parenchymal liver damage manifested by elevated levels of bilirubin concentrations, as well as increased alanine aminotransferase (ALT), aspartate aminotransferase (AST), alkaline phosphatase (ALP), and *γ*-glutamyl transpeptidase activity in the plasma [15].

Surprisingly, plasmodial vacuolar iron transporter (VIT) proteins have been elucidated in *P. falciparum* (called PfVIT) and *P. berghei* (called PbVIT) to detoxify or mobilize labile iron, particularly Fe^2+^ in the red cell cytosol. Iron chelators, including desferrioxamine (DFO), *N*-terminal derivatives of DFO, desferrithiocin, deferiprone (DFP), and dexrazoxane, have been identified as antimalarial agents in *P. falciparum* cultures, blood, and liver stages of *P. berghei*- and *P. yoelii*-infected rodents when targeting chelatable labile and ferritin iron in erythrocyte cytosol and parasite food vacuoles [16–19]. Resveratrol (RVT) is an antioxidative polyphenol that is present in the skin of grapes and is abundant in red wine. Interestingly, RVT derivatives obtained from *Pleuropterus ciliinervis* extracts exerted antimalarial properties in *P. berghei*-infected mice [20]. Likewise, the ethanolic extract of *Mezoneuron benthamianum* Bail leaves was comprised of several phenolic compounds, including RVT, that have effectively exhibited an inhibitory effect on the growth of *P. falciparum* (chloroquine-sensitive strain) [20]. However, RVT was not able to extend the life span of the *Anopheles stephensi* mosquito, which is known to be a vector of human malaria [21]. In theory, this iron chelator could be a potential chemotherapeutic agent due to its ability to withhold available iron and consequently inhibit the growth of the malaria parasite [22, 23]. For multitarget directed ligands, a deferiprone-resveratrol hybrid compound (DFP-RVT) was synthesized by merging DFP with RVT via the established method previously described by Li, et al. [24]. Accordingly, the molecule is comprised of the bidentate iron-chelating part of DFP and the antioxidant part of RVT as is shown in Figure 1.

Recently, we have demonstrated the inhibitory effects of the DFP-RVT hybrid on parasite growth in both *P. falciparum* cultures and *P. berghei*-infected mice. Furthermore, we have reported on the ability of this hybrid to potentially reduce the labile iron pool and oxidative stress in malaria-infected mice [25, 26]. In the present study, we have assessed the hepatoprotective effect of DFP-RVT on *P. berghei*-infected mice.

## 2. Materials and Methods

### 2.1. Chemicals and Reagents

Accordingly, 1-butanol, butylated hydroxytoluene (BHT), dimethyl sulfoxide (DMSO), heme iron reagent, pyrimethamine (PYR), 1, 1, 3, 3-tetramethoxypropane (TMP), thiobarbituric acid (TBA), and Wright−Giemsa staining solution were purchased from Sigma-Aldrich Chemicals, Company (St. Louis, MO, USA). DFP (1, 2-dimethyl-3-hydroxypyridin-4-one) was provided by the Institute of Research and Development, Government Pharmaceutical Organization, Bangkok, Thailand. Enzyme assay kits for AST, ALT, and ALP, along with a colorimetric assay reagent for albumin, were purchased from BIOLABO (Les Hautes Rives, Maizy, France).

### 2.2. Synthesis of DFP-RVT Hybrid

The design, synthesis, and biological evaluation of a series of DFP-RVT compounds were previously described by Li and coworkers [24]. DFP-RVT was labeled with the chemical name 2-(3, 5-dihydroxystyryl)-5-hydroxy-1-methylpyridin-4(1H)-one and the chemical formula C_14_H_14_BrNO_4_ (MW = 340 g/mol).

### 2.3. Animal Ethics

The protocol for animal experimentation was approved by the Institutional Animal Ethics Committee of Walailak University, Thailand (Study Code: WU−AICUC−64013).

### 2.4. Animal Care

Male ICR mice (body weight of approximately 30 g) were purchased from Nomura Siam International Company (Limited), Bangkok, Thailand. The mice were housed separately in polyethylene cages with free access to feed and clean drinking water under controlled conditions of temperature (20–22°C), humidity (50 ± 10%), and light (12 h light/dark cycle). They were acclimatized for one week before experimentation and fed a normal diet (Mouse Feed Food Number CP082, Charoen Pokphand Company, Bangkok, Thailand) containing 495.3 g of carbohydrates, 83.7 g of fat, 269.0 g of protein, 65.4 g of vitamins, and 34.3 g of fiber per 1 kg of feed throughout the course of this study.

### 2.5. *Plasmodium berghei*-Infection in Mice

The rodent malaria parasite, *P. berghei* ANKA strain (PbANKA), was obtained from the Malaria Research and Reference Reagent Resource Center (MR4), Manassas, VA, USA. Cryopreserved parasitized red blood cells (pRBC) were passaged at least once through ICR mice before initiation of the experiment. Parasite growth was monitored daily through analysis of tail vein blood using the Giemsa staining microscopic method. The percentage of parasite growth (% parasitemia) was calculated using the following formula:

(1) $$\begin{array}{c} \%\;parasitemia=\left(number\;of\;pRBC/total\;number\;of\;RBC\right)\times 100\text{.} \end{array}$$

When the % parasitemia reached 15−20%, mouse heart blood was collected in a lithium heparin-coated tube and diluted in 5 mM phosphate buffer saline pH 7.0 (PBS) solution to achieve approximately 1 × 10^7^ pRBC for further passages of the infection in the experiment.

### 2.6. Drug Treatment of PbANKA-Infected Mice

Stock solutions of PYR, DFP, and DFP-RVT were freshly prepared in 100% DMSO. Working doses of the drugs measured in units of mg/kg were adjusted with 60% (*v*/*v*) DMSO. The PbANKA-infected blood (1 × 10^7^ RBC) was injected intraperitoneally into ICR mice. The infected mice were then randomly divided into four groups (3 mice each) and orally administered with 60% DMSO, PYR (2 mg/kg), DFP (50 mg/kg), and DFP-RVT (50 mg/kg) for 8 consecutive days. Mice were then monitored daily in terms of % parasitemia by analysis of tail vein blood using the Giemsa staining microscopic method as has been previously described [25]. The percentage of parasite growth inhibition (%inhibition) was then calculated by using the following formula:

(2) $$\begin{array}{c} \%Inhibition=\left(\%{parasitemia}_{DMSO}-\%{parasitemia}_{Treatment}\times 100\right)/\;\%{parasitemia}_{Treatment}\text{.} \end{array}$$

Mice were sacrificed on day 8 and heart blood was collected for hematological and biochemical analysis. The liver was then removed, weighed, and kept at −80°C for further analysis. The liver weight index (WI) was calculated by dividing the weight by the body weight (BW) of the mice.

### 2.7. Hematological Parameter Measurement

Complete blood counts, including RBC numbers, Hb concentrations, hematocrit (Hct) concentrations, mean corpuscular volume (MCV), mean corpuscular hemoglobin (MCH) concentrations, mean corpuscular hemoglobin concentrations (MCHC), white blood cell (WBC) numbers, and percentage of differential WBC, were determined using an Automatic Cell Counter (Beckman Coulter Life Sciences, Indiana, IN, USA) at the Medical Technology Laboratory, Walailak University, Thailand.

### 2.8. Measurement of Liver Enzyme Activity

AST, ALT, and ALP activities were determined using the specified reagent assay kits (Roche Company, Mannheim, Germany) according to the manufacturer's instructions.

### 2.9. Determination of Heme Concentrations

Heme concentrations were determined in the plasma and liver homogenate using both the heme assay method [3] and the appropriate assay kit according to the manufacturer's instructions.

### 2.10. Measurement of Lipid-Peroxidation Product

In principle, a lipid-peroxidation product, such as malondialdehyde (MDA), reacted with the TBA reagent to form a pink-colored thiobarbituric acid reactive substance (TBARS) [27]. In the assay, plasma and liver homogenates were deproteinized using a solution comprised of 10% (*w*/*v*) trichloroacetic acid (TCA) and 50 mg/L (*w*/*v*) BHT. The homogenates were then centrifuged at 1,500 rpm. The supernatant was collected and incubated with a reaction mixture containing 0.44M H_3_PO_4_ and 0.6% (*w*/*v*) TBA at 90°C for 30 min. The supernatant was then allowed to cool down to 4°C over a period of 10 min. Afterwards, 1-butanol was added in order to extract the pink-colored TBARS from the solution, while optical density (OD) was photometrically measured at 540 nm against the reagent blank. Concentrations of TBARS were determined from a calibration curve of TMP established from a range of different concentrations.

### 2.11. Pathological Examination

Liver tissue samples collected from mice were fixed in 10% (*v*/*v*) formalin at room temperature for 24−48 h. The tissue samples were embedded in paraﬃn and sliced into 5 *µ*m thick sections using a manual rotary microtome (Thermo Scientific™, Germany). They were then processed for the purposes of sequential dehydration and stained with hematoxylin and eosin (H&E) dye using a Gemini AS automated slide staining machine (Thermo Scientific™, Germany). Histopathological changes were examined under a light microscope by an expert pathologist who was blinded to the experimental groups.

### 2.12. Statistical Analysis

Graphs were prepared using the GraphPad Prism version 8.0 Program (GraphPad Prism Software, San Diego, CA, USA). Data were analyzed and expressed as mean ± standard error of the mean values (SEM). Statistical significance was determined using one-way analysis of variance (ANOVA) with posthoc Tukey-Kramer, where the value of *p*  <  0.05 was considered a significant difference.

## 3. Results

### 3.1. Antimalarial Activity of DFP-RVT against PbANKA Infection

As shown in Figure 2, a large number of *P. berghei*-infected RBC were illustrated in mice treated with 60% DMSO (a), while the pRBC were decreased dramatically by PYR treatment (b), moderately by DFPRVT (d) and DFP (c). The percentage of parasite growth in PbANKA-infected mice treated with 60% DMSO was 14.2% when compared with that of uninfected mice (*p*  <  0.05). Accordingly, it decreased dramatically by PYR and DFP-RVT treatment (0.2% and 12.5%, respectively) (*p*  <  0.05) and slightly decreased by DFP treatment (13.5 %) (Figure 3(a)). With regard to the inhibitory effect, PYR completely suppressed the growth of PbANKA (100% inhibition, *p*  <  0.01) in the infected mice, while DFPRVT was moderately suppressed at 26.1% (*p*  <  0.05) and DFP was slightly depressed at 14.1% when compared with the infected group that had been treated with DMSO (Figure 3(b)).

### 3.2. Body, Liver Weight, and Liver Weight Index of PbANKA-Infected Mice

As shown in Figures 4(a) and 4(b), the BW of healthy mice increased over the course of the study. During 8-day PbANKA infection, BW values of the infected groups decreased after treatment with DMSO (control) and DFP (−5.40% and −0.55%, respectively) but increased after treatment with DFP-RVT and PYR (0.54% and 3.98%, respectively). Additionally, the liver weight was found to increase in mice in the PbANKA-infected group that had been treated with DMSO when compared with the normal group (*p*  <  0.05); however, this value was considerably decreased after treatment with PYR or DFP-RVT (*p*  <  0.05) and decreased nonsignificantly after treatment with DFP when compared with the DMSO treatment group (Figure 4(c)). Likewise, the resulting liver WI values were consistent with those of the weight of the liver (Figure 4(d)). These results imply that malaria parasite infection may delay the growth and liver health of the hosts, while DFP-RVT and PYR treatments could restore the liver pathophysiology of the infected hosts.

### 3.3. Hematological Parameter Levels in PbANKA-Infected Mice

In our findings, PbANKA-infected mice exposed to the DMSO treatment showed a significant decrease in RBC numbers, Hb concentrations, and Hct values when compared with normal mice (*p*  <  0.05). Importantly, the PYR (2 mg/kg) treatment of mice in the PbANKA-infected group restored the decrease in RBC indices (*p*  <  0.05), while DFP-RVT (50 mg/kg) treatment did so slightly and the DFP (50 mg/kg) treatment did not influence these values when compared with the DMSO group (Table 1). Among the RBC indices, the MCV values were significantly increased in all of the infected groups when compared to the normal group. This would indicate the presence of macrocytic RBC during malaria infection, while all the treatments significantly reduced the increasing MCV values. With regard to WBC indices, increases in WBC numbers and % neutrophils were observed along with a decrease in % lymphocytes in the PbANKA-infected group treated with DMSO when compared with the normal group (*p*  <  0.05) (Table 2). Surprisingly, the PYR (2 mg/kg) treatment of the infected mice decreased WBC numbers (*p*  <  0.05) and tentatively restored the altered WBC indices, while DFP-RVT (50 mg/kg) reduced WBC numbers (*p*  <  0.05) and slightly changed the differential WBC pattern when compared with the DMSO group. Nevertheless, the DFP (50 mg/kg) treatment had a minimal effect on WBC indices.

### 3.4. Plasma Liver Enzyme Activity of PbANKA-Infected Mice

As is shown in Table 3, levels of plasma AST and ALP (*p*  <  0.05), along with ALT levels, increased in mice in the PbANKA-infected group exposed to the DMSO treatment. Notably, levels of all of the increasing enzymes were restored in the PYR-treated PbANKA infection group (*p*  <  0.05 for ALP), while levels of ALT and ALP were decreased in the DFP-RVT treatment group (*p*  <  0.05). Only the ALP level decreased in the DFP treatment group (*p*  <  0.05) when compared with those of the DMSO treatment group.

### 3.5. Plasma and Hepatic Heme Concentrations of PbANKA-Infected Mice

As a consequence of severe hemolysis during malaria infection, heme-iron levels can be employed to predict the oxidant iron-catalyzed production of ROS, which is known to be harmful to certain tissues and vital organs, particularly the liver. Accordingly, plasma heme concentrations were elevated in PbANKA-infected mice treated with DMSO when compared with normal mice, while the increasing plasma heme decreased significantly after treatments with PYR (2 mg/kg), DFP (50 mg/kg), and DFP-RVT (50 mg/kg) (Figure 5(a)). Consistently, hepatic heme content was significantly increased in the PbANKA-infected mice treated with DMSO when compared with normal mice, while the increasing value was significantly decreased by all three treatments (Figure 5(b)). Taken together, the potency is presented as follows: DFP-RVT > DFP > PYR, suggesting the possible mechanism of this effect would likely be the iron-chelating activity.

### 3.6. Levels of Plasma and Hepatic TBARS in PbANKA-Infected Mice

In fact, redox iron and heme iron levels can potentially be employed to catalyze the generation of ROS, which consequently induces a chained-peroxidation of polyunsaturated fatty acids on cell membranes and plasma lipoproteins. Here, the results indicate that the level of plasma TBARS was significantly increased in PbANKA-infected mice when compared with normal mice. Accordingly, the increasing plasma TBARS levels in PbANKA-infected mice decreased significantly by DFP (50 mg/kg) and decreased slightly by PYR (2 mg/kg) and DFP-RVT (50 mg/kg) treatments (Figure 6(a)). Similarly, levels of hepatic TBARS were significantly increased in the PbANKA infection group when compared with the normal group, while the increasing levels were diminished by all three treatments (Figure 6(b)).

### 3.7. Pathological Illustration of PbANKA-Infected Mice

A microscopic examination of H&E-stained liver sections has revealed that the liver of normal mice showed normal polygonal hepatocytes with acidophilic cytoplasm and normal architecture of the central vein and sinusoids (Figure 7(a)). In contrast, the livers of PbANKA-infected mice indicated areas of hepatocyte necrosis (Figure 7(b), symbol *∗*) and a large number of Kupffer cell infiltrations within sinusoids (Figure 7(b), symbol K). Interestingly, treatment of PbANKA-infected mice with PYR (2 mg/kg) indicated a normal architecture of hepatocytes and the central vein, while a small number of Kupffer cell infiltrations were observed (Figure 7(c)). Surprisingly, treatment of the infected mice with DFP (50 mg/kg) demonstrated normal morphology of hepatocytes and central veins (Figure 7(d)), whereas treatment with DFP-RVT (50 mg/kg) did not decrease the number of presenting Kupffer cells (Figure 7(e)).

## 4. Discussion

Iron plays a crucial role in the cellular metabolism and proliferation of all living organisms including malaria parasites [28]; inversely, the withholding of the available amount of iron from the environment can interfere with the reproduction rates of these organisms [23]. Interestingly, iron-chelating compounds, namely DFO, DFP, *N*-acetyl-6-aminohexyl-3-hydroxy-2-methylpyridin-4-one (or CM1), and (S)-4,5-dihydro-2-(2-hydroxy-4-hydroxyphenyl)-4-methyl-4-thiazolecarboxylic acid polyether, have been reported to be able to inhibit the growth of the *P. falciparum* parasite [22, 23, 29, 30]. In this study, the bidentate iron-chelator hybrid and DFP-RVT exhibited a greater inhibitory effect on *P. berghei* ANKA growth in infected mice than DFP, which is consistent with the degree of antimalarial activity observed in *P. falciparum* cultures [25]. Alternatively, redox iron at the allosteric site of ribonucleotide reductase for DNA synthesis could be another potential target for the antimalarial iron chelator, which is absolutely necessary for many fast-dividing cells including those of bacteria, cancer cells, and malaria parasites [31, 32].

Severe malarial anemia is a secondary consequence of increased RBC hemolysis and erythrophagocytosis. As has been evidenced in this study, *P. berghei* infection resulted in BW and liver weight (also liver WI) losses (possibly due to intestinal parasite infection and liver inflammation), while also resulting in increased MCV and MCH values as well as decreased RDW values (possibly due to reticulocyte compensation and the presence of hemozoin in pRBC). As a result of liver-stage malaria infection, the liver injury will suppress hepcidin production leading to an increase in iron influx from the duodenum and efflux from reticuloendothelial (RE) cells. Consistently, RBC numbers, Hb concentrations, Hct values, and plasma hepcidin concentrations were found to decrease in *P. berghei* K173-infected mice when compared with WT mice [33]. Casals−Pascual and colleagues demonstrated that the hemozoin in parasite food vacuoles and plasma compartments inhibited erythropoiesis and were synergized with the tumor necrotic factor-alpha in this inhibition *in vitro* [34]. Additionally, increased hemolysis occurs at the stage of schizont rupture during malaria infection, which is related to the parasite burden in the body and the acceleration of RBC destruction [3, 35, 36]. According to RBC breakdown, the rupture and phagocytosis of malaria-infected RBC cause severe anemia during the infection. Moreover, the removal of uninfected RBC by IgG sensitization, physicochemical RBC membrane damage, decreasing of erythropoiesis response, malaria infection-induced marrow hypoplasia, increasing of the RE system activity in the spleen, poor nutrition, and intestinal parasite infection were also observed during malaria infection [37–39]. Furthermore, the balance of pro- and anti-inflammatory mediators plays an important role in the inhibition of erythrocyte production (ineffective erythropoiesis) and can cause organ dysfunction [40]. This study has highlighted the determination that DFP-RVT can slightly improve the hematological parameters of RBC production in terms of RBC numbers, Hb concentrations, Hct levels, and MCV values, while PYR completely restored the RBC indices to normal levels. These findings imply that the *P. berghei* parasite burden is correlated to the severity of hemolysis and the improvement of RBC production. With regard to WBC indices, the number of neutrophils in *P. berghei*-infected mice increased, while the number of lymphocytes decreased. In contrast, previous studies have reported that alterations of absolute and differential WBC were associated with the severity of malaria infection and response to the treatment [41, 42]. The phagocytosis activity of neutrophils is the first response to malaria infection, whereas circulating lymphocytes were decreased as a result of the apoptosis response of mononuclear cells in malaria infections [43].

During the erythrocyte stage of malaria infection, pRBC are sequestered in small blood vessels and can induce the impairment of blood flow to the tissue leading to the failure of several organs including the liver [44, 45]. Crucially, intravascular hemolysis in malaria infection increases oxidative stress and the infiltration of leukocytes into the liver tissue, which are known to enhance hepatic inflammation [46]. Pathologically, liver dysfunction is a common manifestation of severe malaria infection. It is known to contribute to several complications, including hypoglycemia and metabolic acidosis [45, 47], which are indicated by liver enlargement and an increase in liver enzymes [48]. In our findings, we have revealed that an elevation of plasma AST, ALT, and ALP activities during *P. berghei* infection would indicate liver damage, while treatments with PYR, DFP, and DFP-RVT considerably restored the increasing liver enzyme activities close to the levels found in healthy mice. Surprisingly, increased liver enzyme activities were found in *P. falciparum* infection and correlated to the sequestration of pRBC in the liver, while they could be restored over 3−6 weeks or after initiation of the treatment [45]. Additionally, the enlargement of the liver was found to be associated with morbidity, whereas hepatomegaly was reported as a common finding in malaria infection [49]. This seems to be correlated with the degree of pRBC sequestration in the liver [48]. Again, monotherapy with PYR and DFP-RVT was effective in retaining the size of the liver during malaria infection. This would suggest that PYR and DFP-RVT possibly decreased the trapping of pRBC in the liver.

The hemolysis of RBC that occurs in malaria parasite infection results in the release of heme, a toxic pro-oxidant that is degraded by heme oxygenase 1 (HO−1) [50]. It is apparent that iron and heme are essential nutrients for fast-dividing pathogenic organisms; on the contrary, the control of labile heme is a crucial strategy for the survival of the malaria parasite [51]. Generally, heme in the blood circulation is cleared by the protein hemopexin, which is then taken up by hepatocytes. Once the hemolysis becomes severe and persistent, the hemopexin fails to counteract the high number of free hemes circulating in the blood. Under unusual conditions, the iron in the heme molecule could generate ROS via the Fenton reaction causing oxidative tissue damage and cell death [52]. In the present study, we found that the infection of PbANKA increased the levels of heme in both plasma and liver tissues, which were correlated with the levels of the MDA product represented by TBARS concentrations. The histopathological liver tissue was indicative of the necrosis area, which would indicate the oxidative tissue damage that occurs from ROS. These outcomes would be consistent with the findings of a previous study reporting on liver necrosis in *P. falciparum*-infected patients [53, 54]. Fortunately, the treatment of PbANKA-infected mice with PYR, DFP, and DFP-RVT significantly reduced the levels of heme in both plasma and liver tissues, which were relevant to the levels of TBARS concentrations in plasma and liver tissues. Impressively, DFP-RVT showed a better effect than PYR and DFP in terms of a reduction in heme levels. More or less, DFP-RVT exhibited higher lipophilicity than DFP, which would indicate greater accessibility to liver cells and the exertion of potent antioxidant activity [26]. Additionally, the histological feature of the liver tissue was normal when treated with PYR, DFP, and DFP-RVT. Taken together, DFP-RVT exhibited a potentially beneficial effect on the inhibition of malaria parasite growth, restored the erythropoiesis parameters, and mitigated liver inflammation by chelating redox iron and scavenging free radicals in the liver cells.

## 5. Conclusion

Iron is essentially required for plasmodium metabolism and can induce ROS-mediated liver injury in the host. Here, a DFP-RVT hybrid inhibited blood-stage *P. berghei* growth by depriving heme iron utilization and mitigating liver injury through the inhibition of iron-catalyzed lipid peroxidation. Altogether, our DFP-RVT hybrid potentially exerted parasite-inhibitory and hepatoprotective effects during malaria infection. The degree of efficacy, as well as that of toxicity, for the combined treatments of DFP-RVT and antimalarial drugs at therapeutic doses should be further evaluated in *in vivo* studies.

## Figures and Tables

**Figure 1:** Chemical structure of DFP-RVT hybrid (redrawn from [25]).

**Figure 2:** Blood film of PbANKA infection in mice treated with DMSO (a), PYR (b), DFP (c), and DFPRVT (d). Male ICR mice (*n* = 3 each) were intraperitoneally infected with pRBC suspension (approximately 1 × 10^7^ cells/mL with 10−20% parasitemia) and orally administered with 60% DMSO, PYR (2 mg/kg BW), DFP (50 mg/kg BW), and DFP-RVT (50 mg/kg BW) everyday for 8 consecutive days. Blood-stage percentage of pRBC was determined using the microscopic Giemsa staining method. BW = body weight, DFP = deferiprone, DFP-RVT = deferiprone-resveratrol, DMSO = dimethylsulfoxide, PbANKA = *P. berghei* ANKA strain, pRBC = parasitized red blood cell, and PYR = pyrimethamine.

**Figure 3:** Antimalarial activity of DFP-RVT, DFP, and PYR in PbANKA-infected mice. The PbANKA-infected mice were orally administered with 60% DMSO, PYR (2 mg/kg BW), DFP (50 mg/kg BW), and DFP-RVT (50 mg/kg BW) everyday for 8 consecutive days. The percentage of pRBC was determined using the microscopic Giemsa staining method and presented as either % parasitemia (a) or % suppression (b). Data are expressed as mean ± SEM values. Accordingly, ^#^*p*  <  0.05 when compared with the uninfected PbANKA group; and ^*∗*^*p*  <  0.05, ^*∗∗*^*p*  <  0.01 when compared with the infection group treated with DMSO. BW = body weight, DFP = deferiprone, DFP-RVT = deferiprone-resveratrol, DMSO = dimethylsulfoxide, PbANKA = *P. berghei* ANKA strain, pRBC = parasitized red blood cell, PYR = pyrimethamine, and SEM = standard error of mean values.

**Figure 4:** BW (a), % BW change (b), liver weight (c), and liver WI (d) of normal mice and PbANKA-infected mice treated with 60% DMSO, DFP-RVT (50 mg/kg BW), DFP (50 mg/kg BW), and PYR (2 mg/kg BW) for 8 consecutive days. Data are expressed as mean ± SEM values (*n* = 3 each). Accordingly, ^#^*p*  <  0.05 when compared with the normal group; and ^*∗*^*p*  <  0.05 when compared with the PbANKA-infected group treated with DMSO. BW = body weight, DFP = deferiprone, DFP-RVT = deferiproneresveratrol, DMSO = dimethylsulfoxide, PbANKA = *P. berghei* ANKA strain, pRBC = parasitized red blood cell, PYR = pyrimethamine, SEM = standard error of the mean values, and WI = weight index.

**Figure 5:** Heme iron concentrations of the plasma (a) and liver (b) of normal mice and *Pb*ANKA-infected mice treated with 60% DMSO, DFP-RVT (50 mg/kg BW), DFP (50 mg/kg BW), and PYR (2 mg/kg BW) for 8 consecutive days. Data are expressed as mean ± SEM values (*n* = 3 each). Accordingly, ^#^*p*  <  0.05 when compared with the normal group; and ^*∗*^*p*  <  0.05 when compared with the PbANKA-infected group treated with DMSO.

**Figure 6:** Levels of TBARS in the plasma (a) and liver (b) of normal mice and PbANKA-infected mice (*n* = 3 each) treated with 60% DMSO, DFP (50 mg/kg BW), DFP-RVT (50 mg/kg BW), and PYR (2 mg/kg BW) for 8 consecutive days. Data are expressed as mean ± SEM values. Accordingly, ^#^*p*  <  0.05 when compared with the normal mice; and ^*∗*^*p*  <  0.05 when compared with the PbANKA-infected mice that had been treated with DMSO.

**Figure 7:** Histopathology of H&E-stained liver tissues collected from normal mice (a) and PbANKA-infected mice treated with 60% DMSO (b), DFP (50 mg/kg) (c), DFP-RVT (50 mg/kg) (d), and PYR (2 mg/kg) (e) for 8 consecutive days. H = hepatocyte, S = sinusoid, CV = central vein, K = Kupffer's cell, and ^*∗*^ = necrosis area.

**Table 1:** Hematological parameter levels in normal mice treated with DI and PbANKA-infected mice treated with 60% DMSO, DFP-RVT (50 mg/kg), DFP (50 mg/kg), and PYR (2 mg/kg) (*n* = 3 each) for 8 consecutive days. Data are expressed as mean ± SEM values. Accordingly, ^#^*p*  <  0.05 when compared with the normal group; and ^*∗*^*p*  <  0.05 when compared with the PbANKA-infected group treated with DMSO. (a) RBC indices.

Mice	Treatment	RBC number(×10^6^/mL)	Hb (g/dL)	Hct (%)	MCV (fL)	MCH (pg)	MCHC (g/dL)	RDW (%)
Normal	DI	8.86 ± 0.84	13.45 ± 1.25	45.60 ± 6.20	51.10 ± 1.90	15.25 ± 0.25	29.80 ± 1.80	15.55 ± 0.55
*Pb*ANKA-infected	DMSO	4.74 ± 0.30^#^	8.80 ± 0.65^#^	30.00 ± 1.63^#^	62.33 ± 1.20^#^	18.67 ± 0.33	30.00 ± 0.58	13.33 ± 0.88
*Pb*ANKA-infected	PYR	9.66 ± 0.23^*∗*^	16.10 ± 0.40^*∗*^	54.00 ± 2.08^*∗*^	56.00 ± 1.15^*∗*^	16.67 ± 0.33	29.67 ± 0.67	13.67 ± 0.33
*Pb*ANKA-infected	DFP	4.57 ± 0.27	8.70 ± 0.33	29.50 ± 0.41	65.00 ± 2.45	19.00 ± 0.58	30.33 ± 0.88	13.67 ± 0.88
*Pb*ANKA-infected	DFP-RVT	4.89 ± 0.01	8.50 ± 0.33	26.67 ± 0.67	56.67 ± 2.03^*∗*^	17.67 ± 0.33	31.00 ± 0.58	14.33 ± 0.33

DFP = deferiprone, DFP-RVT = deferiproneresveratrol, DI = deionized water, DMSO = dimethylsulfoxide, Hb = hemoglobin, Hct = hematocrit, MCH = mean corpuscular hemoglobin, MCHC = mean corpuscular hemoglobin concentration, MCV = mean corpuscular volume, PbANKA = *Plasmodium berghei* ANKA strain, PYR = pyrimethamine, RBC = red blood cell, and RDW = red cell distribution width.

**Table 2:** Hematological parameter levels in normal mice treated with DI and PbANKA-infected mice treated with 60% DMSO, DFP-RVT (50 mg/kg), DFP (50 mg/kg), and PYR (2 mg/kg) (*n* = 3 each) for 8 consecutive days. Data are expressed as mean ± SEM values. Accordingly, ^#^*p*  <  0.05 when compared with the normal group; and ^*∗*^*p*  <  0.05 when compared with the PbANKA-infected group treated with DMSO. (b) WBC indices.

Mice	Treatment	WBC number (×10^3^/mL	Differential number (%)				
			Neutrophil	Lymphocyte	Monocyte	Basophil	Eosinophil
Normal	DI	3.10 ± 0.29	17.00 ± 5.00	80.00 ± 6.00	4.00 ± 0.01	ND	ND
*Pb*ANKA-infected	DMSO	16.22 ± 2.10^#^	49.67 ± 3.33^#^	46.33 ± 3.33^#^	2.33 ± 0.33	1.00 ± 0.00	1.00 ± 0.58
*Pb*ANKA-infected	PYR	4.05 ± 0.14^*∗*^	35.00 ± 1.63	54.50 ± 3.67	7.67 ± 2.19	1.00 ± 0.00	0.50 ± 0.41
*Pb*ANKA-infected	DFP	11.99 ± 2.40	45.00 ± 3.51	51.33 ± 3.67	2.33 ± 0.33	1.00 ± 0.58	0.33 ± 0.33
*Pb*ANKA-infected	DFP-RVT	11.10 ± 1.73^*∗*^	46.50 ± 9.39	43.33 ± 9.61	3.00 ± 0.58	0.67 ± 0.33	0.67 ± 0.67

DFP = deferiprone, DFP-RVT = deferiproneresveratrol, DI = deionized water, DMSO = dimethylsulfoxide, ND = not detectable, PbANKA = *Plasmodium berghei* ANKA strain, and PYR = pyrimethamine.

**Table 3:** Levels of AST, ALT, and ALP activities in the plasma of normal mice and PbANKA-infected mice treated with 60% DMSO, DFP (50 mg/kg), DFP-RVT (50 mg/kg), and PYR (2 mg/kg) (*n* = 3 each) for 8 consecutive days. Data are expressed as mean ± SEM values. Accordingly, ^#^*p*  <  0.05 when compared with the normal group; and ^*∗*^*p*  <  0.05 when compared with mice in the PbANKA-infected group that had been treated with DMSO.

Mice	Treatment	Liver enzyme activity		
		AST (U/L)	ALT (U/L)	ALP (U/L)
Normal	DI	51.0 ± 1.4	25.6 ± 1.2	25.3 ± 0.4
*Pb*ANKA-infected	DMSO	81.7 ± 0.7^#^	35.8 ± 2.2	45.8 ± 0.1^#^
*Pb*ANKA-infected	PYR	68.5 ± 4.0	25.7 ± 3.7	30.0 ± 0.5^*∗*^
*Pb*ANKA-infected	DFP	102.8 ± 3.7	36.2 ± 1.1	28.5 ± 0.3^*∗*^
*Pb*ANKA-infected	DFP-RVT	80.8 ± 0.1	20.6 ± 0.6^*∗*^	30.5 ± 1.4^*∗*^

ALP = alkaline phosphatase, ALT = alanine aminotransferase, AST = aspartate aminotransferase, DFP = deferiprone, DFP-RVT = deferiproneresveratrol, DI = deionized water, DMSO = dimethylsulfoxide, PbANKA = *Plasmodium berghei* ANKA strain, and PYR = pyrimethamine.

## Data Availability

The authors confirm that the data supporting the findings of this study are available within the article. In addition, the data are available upon request submitted to Hataichanok Chuljerm.

## Abbreviations/Symbols

ALT: Alanine aminotransferase
ANOVA: One-way analysis of variance
ALP: Alkaline phosphatase
ALT: Alanine aminotransferase
AST: Aspartate aminotransferase
BHT: Butylated hydroxytoluene
BW: Body weight
CV: Central vein
DFO: Desferrioxamine
DFP: Deferiprone or 1, 2-dimethyl-3-hydroxypyridin-4-one
DFP-RVT: Deferiprone−resveratrol hybrid or 2-(3, 5-dihydroxystyryl)-5-hydroxy-1-methylpyridin-4(1H)-one
DMSO: Dimethyl sulfoxide
H: Hepatocyte
Hb: Hemoglobin
Hct: Hematocrit
H&E: Hematoxylin and eosin
HO: Heme oxygenase
HO−1: Heme oxygenase 1
K: Kupffer's cell
CV: Mean corpuscular volume
MCH: Mean corpuscular hemoglobin
MCHC: Mean corpuscular hemoglobin concentration
MDA: Malondialdehyde
OD: Optical density
PbANKA: *Plasmodium berghei* ANKA strain
PBS: Phosphate buffer saline
pRBC: Parasitized red blood cells
PYR: Pyrimethamine
RBC: Red blood cell
ROS: Reactive oxygen species
RE: Reticuloendothelial
RVT: Resveratrol
S: Sinusoid
TBA: Thiobarbituric acid
TBARS: Thiobarbituric acid reactive substance
TCA: Trichloroacetic acid
TMP: 1, 1, 3, 3-tetramethoxypropane
VIT: Vacuolar iron transporter
WBC: White blood cell
WI: Weight index.
